# Impaired GABA_B_-mediated presynaptic inhibition increases excitatory strength and alters short-term plasticity in synapsin knockout mice

**DOI:** 10.18632/oncotarget.21405

**Published:** 2017-09-30

**Authors:** Pierluigi Valente, Pasqualina Farisello, Flavia Valtorta, Pietro Baldelli, Fabio Benfenati

**Affiliations:** ^1^ Department of Experimental Medicine, Section of Physiology, University of Genoa, 16132 Genova, Italy; ^2^ Center for Synaptic Neuroscience and Technology, Istituto Italiano di Tecnologia, 16132 Genova, Italy; ^3^ S. Raffaele Scientific Institute and Vita-Salute University, 20132 Milano, Italy

**Keywords:** epilepsy, excitatory transmission, GABA receptors, facilitation, synaptic depression

## Abstract

Synapsins are a family of synaptic vesicle phosphoproteins regulating synaptic transmission and plasticity. *SYN1/2* genes are major epilepsy susceptibility genes in humans. Consistently, synapsin I/II/III triple knockout (TKO) mice are epileptic and exhibit severe impairments in phasic and tonic GABAergic inhibition that precede the appearance of the epileptic phenotype. These changes are associated with an increased strength of excitatory transmission that has never been mechanistically investigated. Here, we observed that an identical effect in excitatory transmission could be induced in wild-type (WT) Schaffer collateral-CA1 pyramidal cell synapses by blockade of GABA_B_ receptors (GABA_B_Rs). The same treatment was virtually ineffective in TKO slices, suggesting that the increased strength of the excitatory transmission results from an impairment of GABA_B_ presynaptic inhibition. Exogenous stimulation of GABA_B_Rs in excitatory autaptic neurons, where GABA spillover is negligible, demonstrated that GABA_B_Rs were effective in inhibiting excitatory transmission in both WT and TKO neurons. These results demonstrate that the decreased GABA release and spillover, previously observed in TKO hippocampal slices, removes the tonic brake of presynaptic GABA_B_Rs on glutamate transmission, making the excitation/inhibition imbalance stronger.

## INTRODUCTION

Synapsins (Syns) are a family of synaptic vesicle (SV)-associated phosphoproteins that play multiple roles in neural development, synaptic transmission and plasticity. The Syn family is composed of three gene products (Syn I, Syn II and Syn III) that exist in multiple splice isoforms. Syns interact with SVs and actin and regulate SV trafficking and availability for release at both pre- and post-docking steps of exocytosis [1].

Constitutive deletion of one or more Syn genes, with the notable exception of the single deletion of *SYN3*, generates a temporal lobe-like epileptic phenotype characterized by partial, secondarily generalized tonic-clonic seizures starting after the first two months of life and increasing in severity with age and with the number of inactivated Syn genes [2–4] (see [5, 6] for review). Rarely spontaneous, seizures are more frequently evoked by sudden or novel sensory stimuli and are followed by a post-ictal period with typical harmonic oscillations in the EEG during which the animal is completely immobile [7–9].

Interestingly, several loss-of-function mutations in *SYN1* and *SYN2* genes have been identified in patients suffering of epilepsy and/or autism spectrum disorders (ASD) [10–15] and *SYN2* has been identified as one of the highest risk epilepsy genes in a wide screen population [16]. To confirm the reliability of the mouse knockout (KO) models in reproducing the human disease, patients harboring *SYN1* mutations display reflex seizures triggered by sensory stimuli (reflex epilepsy; [15]), while Syn I and Syn II KO mice display various behavioral traits of ASD [17, 18].

Several studies have attempted to clarify the synaptic phenotype of Syn KO mice. In mice, the absence of either Syn I or Syn II primarily affects γ-aminobutyric acid (GABA) transmission, albeit in a different fashion. In hippocampal and cortical neurons of Syn I KO mice, synchronous GABA transmission is selectively impaired [19, 20] while, in hippocampal slices of Syn II KO mice, the asynchronous GABA release is virtually abolished [21], resulting a in a marked decrease in tonic inhibition [22]. Triple Syn I/II/III KO (TKO) mice recapitulate the phenotype of the single Syn I and Syn II KO mice. Indeed, in TKO hippocampal slices, an impaired phasic GABAergic transmission was accompanied by a parallel lower tonic inhibition [4, 23]. This loss-of-function phenotype was surprisingly associated with an increased strength of excitatory transmission observed in both Syn I KO primary autaptic neurons [20] and hippocampal slices of TKO mice [23]. Such increase in excitatory transmission, together with the impairment of GABAergic inputs is at the basis of a strong excitation/inhibition (E/I) imbalance that is responsible for epileptogenesis during the pre-symptomatic period [23–25].

As Syns act by increasing SV availability and facilitating the post-docking stages of release at the nerve terminal level [1], the increased basal glutamatergic transmission cannot be easily explained as a primary synaptic consequence of Syn deletion. Since presynaptic GABA_B_ receptors (GABA_B_Rs) present on glutamatergic terminals and stimulated by extracellular GABA [26] are known to negatively modulate glutamate release [27, 28] and play a role in epileptogenesis (see [29–32] for review), we addressed the possibility that the increase in excitatory strength is due, al least in part, to a dysfunction of the presynaptic GABA_B_ receptor (GABA_B_R)-mediated brake on glutamate release. We compared the effects of specific GABA_B_R antagonists and agonists ((2S)-3-[[(1S)-1-(3,4-dichlorophenyl) ethyl] amino-2-hydroxypropyl] (phenylmethyl) phosphinic acid (CGP55845) and baclofen, respectively) on excitatory synaptic transmission and short-term plasticity in hippocampal slices and primary hippocampal neurons. We found that the glutamatergic phenotype is largely attributable to a lack of tonic activation of presynaptic GABA_B_Rs because of the low extracellular GABA. These findings clarify the molecular mechanisms underlying the epileptic phenotype observed in TKO mice as well as in humans carrying loss-of-function mutations in Syn genes and suggest novel therapeutic approaches for the correction of the E/I imbalance that triggers epileptogenesis.

## RESULTS

### Blockade of GABA_B_ receptors is ineffective in modulating basal glutamatergic transmission in the hippocampal slices from TKO mice

We analyzed evoked release of glutamate from Schaffer collaterals to CA1 pyramidal neurons in acute hippocampal slices from 1-month-old TKO (i.e. before the appearance of the first signs of epilepsy) and in slices from age-matched wild type (WT) mice. Schaffer collaterals were stimulated at increasing intensities (from 10 to 80 μA) and the evoked excitatory postsynaptic current (eEPSC) amplitude was plotted against the stimulation intensity.

Consistent with previous results [23], excitatory synapses from TKO mice exhibited eEPSCs with higher amplitudes in response to the same stimulation intensities than excitatory synapses from age-matched WT mice (Figure 1A and 1B). Potential mechanisms for the enhanced excitatory strength could consist of impaired expression, functioning or activation of presynaptic GABA_B_Rs that act by reducing glutamate release from excitatory terminals [27, 31]. Thus, we tested the possibility that the increased strength of glutamatergic transmission is a consequence of a change in the tonic activation of presynaptic GABA_B_Rs by extracellular GABA, by applying the specific GABA_B_R blocker CGP55845 (5 μM).

**Figure 1:** GABA_B_R blockade with CGP55845 modulates evoked eEPSCs at Schaffer collaterals/CA1 pyramidal neuron synapses of WT, but not TKO, hippocampal slices **(A**, **B)** Effects of increasing stimulation intensities on eEPSC amplitudes in CA1 pyramidal neurons from WT (A) and TKO (B) mice in the absence (black trace/symbols) or presence (red trace/symbols) of 5 μM CGP55845. eEPSCs were evoked in pyramidal neurons by electrical stimulation of Schaffer collaterals. The plots show the effects of GABA_B_R block by CGP55845 on the eEPSC amplitude in the two genotypes. Data are plotted as mean (± sem) current amplitude *versus* stimulation intensity. Representative eEPSC traces evoked in WT and TKO pyramidal neurons in the absence (black) or presence (red) of CGP55845 are reported. **(C)** Comparison of the mean (± sem) eEPSC amplitude evoked with a 70 μA stimulation as a function of the genotype in the absence (left) or presence of CGP55845 (right). Data were analyzed by the unpaired Mann-Whitney's *U*-test; ^*^p<0.05; ^**^p<0.01. WT: n=9 and n=5; TKO: n=9 and n=5; for vehicle and CGP, respectively.

Interestingly, while the application of CGP55845 significantly increased glutamatergic transmission in WT slices, particularly at high stimulation intensities (Figure 1A), it was virtually ineffective in further increasing the potentiated glutamatergic transmission of TKO slices (Figure 1B). The analysis of the effect of the genotype revealed that the GABA_B_R blocker attenuated the difference in eEPSC amplitude between WT and TKO slices (Figure 1C), as a consequence of the total lack of effect of CGP55845 in the TKO background.

These results demonstrate that, in TKO mice, the presynaptic GABA_B_R-mediated inhibition of the eEPSC is virtually absent, providing a possible explanation for the enhancement of excitatory synaptic transmission associated with deletion of the three Syn genes.

### Enhanced synaptic depression of TKO Shaffer-CA1 synapses is due to the lack of GABA_B_R presynaptic inhibition

We previously demonstrated that when the Schaffer collateral pathway is stimulated for 20 s at 20 Hz, WT glutamatergic synapses respond to the stimulation with a long-lasting facilitation, while TKO excitatory synapses show only a transient facilitation followed by a profound and sustained depression [23]. Moreover, we have recently shown that, in addition to negatively modulating glutamate release evoked by single pulses, the activation of presynaptic GABA_B_Rs boosts synaptic strength during high frequency stimulation, by switching glutamatergic transmission from a high to low release probability level [33].

Based on these considerations, the Schaffer collateral pathway of WT and TKO mice was stimulated with a train of 400 stimuli delivered at 20 Hz in the presence of CGP55845 (5 μM; Figure 2A). In agreement with previous reports [33, 34], the blockade of GABA_B_Rs had a striking effect on WT glutamatergic synapses: facilitation was markedly inhibited, except for a very early period in the train, and was replaced by a profound depression that, however, had slower kinetics than that experienced by TKO neurons (Figure 2B, left panel). Strikingly, application of CGP55845 was totally ineffective in modulating the response of TKO neurons to high frequency stimulation (Figure 2B). This result suggests that a lack of GABA_B_R-mediated presynaptic inhibition contributes to the sustained synaptic depression that characterizes TKO synapses under basal conditions.

**Figure 2:** GABA_B_R blockade greatly increased depression at Schaffer collaterals/CA1 pyramidal neuron synapses of WT, but not TKO, hippocampal slices **(A)**, **(B)** Effects of sustained and high frequency stimulation of Schaffer collaterals (20 s at 20 Hz) in CA1 pyramidal neurons from WT (left) and TKO (right) mice in the absence (black traces/symbols) or presence (red traces/symbols) of CGP55845. A sustained facilitation was present in WT mice, which became transient and associated with late depression in the presence of CGP. On the contrary, the profound depression following a short-lived facilitation observed in TKO mice was unaffected by CGP. Representative traces of eEPSCs in response to the 1^st^, 2^nd^ and last action potential in the train are shown, normalized to the amplitude of the first response (WT, 97.9 pA; WT+CGP, 249.6 pA; TKO, 430.2 pA; TKO+CGP, 408.0 pA) (A). In the main plots, the amplitude of eEPSCs, normalized to the mean baseline value is plotted as a function of time (B). **(C)** Mean (± sem) percentage of depression of eEPSC amplitude as a function of the genotype in the absence (left; black bars) or presence of CGP55845 (right; red bars). Quantitative analysis of depression was carried out by measuring the first eEPSC 0.5 s after the peak of facilitation (I_p_) and 10 s after the start of the train stimulation (I_10 s_), according to the formula: (I_p_-I_10s_)/I_p_^*^100 (see panel B). The effects of GABA_B_R block by CGP55845 in the two genotypes were analyzed using the unpaired Mann-Whitney's *U*-test; ^*^p<0.05; ^**^p<0.01. **(D)**, **(E)** The time course of recovery, studied for 600 s after the end of the train by lowering the stimulation frequency from 20 to 0.1 Hz, is shown for WT (left) and TKO (right) slices in the absence (black) or presence (red) of CGP55845. Representative traces of eEPSCs at various times of recovery are shown after normalization to the baseline (bsl) amplitudes (WT, 87.5 pA; WT+CGP, 239.4 pA; TKO, 427.1 pA; TKO+CGP, 400.3 pA) (D). In the main plots, the amplitude of eEPSCs, normalized to the mean baseline value, is plotted as a function of time (E). ^*^p<0.05, #p<0.05, for untreated and CGP-treated samples, respectively; one-tailed paired Student's *t*-test *vs* mean steady-state values calculated in the last 5 min of recording (shaded area). WT, n=11 and n=10; TKO, n=6 and n=10; for vehicle and CGP, respectively.

The analysis of the effect of genotype in the presence of the GABA_B_R blockade (Figure 2C) revealed that the difference in the extent of eEPSC depression between WT and TKO slices was greatly attenuated, as a consequence of the strong depressive effect of CGP55845 in WT slices, as compared to its virtual lack of effect in the TKO background (Figure 2B).

When the stimulation frequency was lowered to 0.1 Hz after the end of the train, the facilitation observed in WT untreated slices, as well as the depression displayed by CGP55845-treated WT slices, were both short-lasting and returned to baseline in 50-60 s (Figure 2D, 2E, left panels). A similar kinetics of recovery from depression, which was not affected by CGP55845 treatment, was observed in TKO slices (Figure 2D, 2E; right panels).

### Exogenous activation of the GABA_B_Rs is preserved in Syn I, Syn II or TKO autaptic neurons

In principle, a lack of effect of the GABA_B_R blockade could be due to either a defective GABA_B_R-mediated transmission or a ceiling effect produced by the Syn mutation that occludes the modulation by GABA_B_Rs. In turn, a defective GABA_B_R-mediated transmission can be due to lack in the expression of GABA_B_Rs on the presynaptic membrane of excitatory neurons, impaired GABA_B_R-linked intracellular signaling or exceedingly low extracellular GABA concentrations. To identify the exact mechanism, we used primary cultures of hippocampal autaptic neurons that, by virtue of their extremely low cell density, allow to precisely control the extracellular medium [20, 35], thus avoiding paracrine effects of released neurotransmitters spilled over from neighboring synapses [33]. Excitatory autaptic neurons, held at −70 mV, were stimulated at 0.1 Hz for over 2 min to obtain a stable baseline before the application of GABA_B_R active drugs (Figure 3A).

**Figure 3:** GABA_B_ receptors are functional in WT, Syn I KO, Syn II KO and Syn TKO hippocampal neurons **(A)** Representative autaptic eEPSCs recorded in WT, Syn I KO, Syn II KO and TKO hippocampal neurons under control conditions (ctrl; black traces) and in the presence of either 20 μM baclofen (Bclf; blue traces) or 5 μM CGP55845 (CGP; red traces). To detect the effects of the GABA_B_R block with CGP55845, eEPSCs were recorded in the presence of GABA (1 μM) in the extracellular solution. Currents were elicited clamping the cell under study at –70 mV and then by stimulating with a step to +40 mV (0.5 ms at 0.1 Hz, inset). Stimulation artifacts were blanked for clarity. **(B)** Mean (± sem) changes in eEPSC amplitude induced by baclofen and CGP55845. The superimposed symbols represent individual eEPSC values before (ctrl or GABA alone) and after treatment with either baclofen (blue bars) or CGP55845 (in GABA; red bars). Data were analyzed by using the two-tailed paired Student's *t*-test; ^**^p<0.01; ^***^p<0.001. **(C)** The mean (± sem) effect of either baclofen (blue bars) or CGP55845 (in GABA; red bars) on eEPSC amplitude across genotypes, shown in percent of the respective effect observed in WT neurons, shows a similar extent of modulation across genotypes. Data, analyzed by one-way ANOVA/Bonferroni's tests, were not significantly different. WT: n=12 and n=11; Syn I KO: n=11 and n=13; Syn II KO: n=11 and n=10; Syn TKO: n= 12 and n=11, for Bclf and CGP treatments, respectively.

To estimate the presence of functional GABA_B_Rs controlling glutamate release from excitatory autaptic terminals, we challenged autaptic neurons with the potent and selective agonist baclofen and the specific antagonist CGP55845. The latter blocker was tested in the presence of 1 μM exogenous GABA to tonically activate GABA_B_Rs. As previously reported [33], baclofen induced an over two-fold decrease in the eEPSC amplitude in WT neurons, while the application of CGP55845 in GABA dramatically increased eEPSC amplitude (Figure 3A, 3B). When the same treatment was applied to Syn I KO, Syn II KO or TKO autaptic neurons, the effects were substantially similar across all genotypes (Figure 3B, 3C). The results demonstrate that functional GABA_B_Rs are correctly expressed in Syn KO neurons and that their affinity for agonists and intracellular signaling are intact.

Presynaptic GABA_B_Rs are known to exert a brake on glutamate release by negatively controlling Ca^2+^ influx, presynaptic depolarization and SV availability for release (see [30] for review). To fully exploit their function, we investigated paired-pulse facilitation, an exquisitely presynaptic form of short-term plasticity that mainly depends on the initial release probability. In WT autapses, baclofen induced a marked, persistent and highly significant facilitation in response to the second pulse with a significant increase in the paired-pulse ratio (PPR), while CGP55845 in the presence of GABA significantly decreased PPR. These effects were qualitatively preserved across genotypes (Figure 4A-4C). As a decrease in the initial release probability is the main drive of facilitation and the predominant effect of GABA_B_R activation, the data indicate that GABA_B_R signaling is functional in Syn KO neurons.

**Figure 4:** Exogenous activation of GABA_B_ receptors similarly affects short-term plasticity of glutamatergic transmission in WT, Syn I KO, Syn II KO and Syn TKO hippocampal autapses **(A)** Paired pulse eEPSCs at 50 ms inter-stimulus interval were recorded in WT, Syn I KO, Syn II KO and TKO hippocampal autapses under control conditions (ctrl; black traces) and in the presence of either 20 μM baclofen (Bclf; blue traces/symbols) or 5 μM CGP55845 (CGP; red traces/symbols). Samples to be challenged with CGP55845 were recorded in the presence of 1 μM GABA in the extracellular solution. Representative paired pulse traces (0.1 Hz, inter-pulse interval 50 ms, inset) are represented without artifact for clarity. **(B)** The time course of the paired-pulse ratio (PPR), calculated as the amplitude ratio between the second to the first response (I_2_/I_1_), is shown as means ± sem for the four genotypes during the 10 min treatment with either baclofen or CGP55845 (in GABA). **(C)** Changes (means ± sem) in PPR induced by baclofen and CGP55845 (in GABA) in WT, Syn I KO, Syn II KO and TKO neurons before (ctrl) and 10 min after the respective treatment. Data were analyzed by using the two-tailed paired Student's *t*-test; ^***^p<0.001. WT: n=9 and n=9; Syn I KO: n=11 and n=11; Syn II KO: n= 10 and n=8; Syn TKO: n=13 and n=13, for baclofen and CGP, respectively.

To better define to what extent GABA_B_R signaling modulates the quantal parameters of synchronous glutamate release, we estimated the readily releasable pool for synchronous release (RRP) and the probability of release of any given SV in the RRP (Pr) using cumulative amplitude analysis. When neurons were challenged with a train of 1.5 s at 40 Hz (60 action potentials), a significant depression of eEPSCs became apparent during the stimulation period irrespective of the amplitude of the first current in the train (Figure 5A). Accordingly, the cumulative profile of the eEPSC amplitude displays a rapid rise followed by a slower linear increase reflecting the equilibrium between depletion and constant replenishment of the RRP (Figure 5B). The graphical extraction of the RRP and Pr from the cumulative curves of individual WT neurons showed that the decrease in the single eEPSC amplitude induced by GABA_B_Rs activation with baclofen is due to a marked drop in Pr and a slighter, but significant, decrease in RRP, while the increase in eEPSC amplitude following blockade of GABA_B_Rs with CGP55845 in GABA elicited a strong increase in Pr accompanied by a slighter, but significant, rise in RRP (Figure 5C). Both effects are believed to contribute to the opposite effects of baclofen and CGP55845 treatments on facilitation, although the changes in Pr are likely to give the larger contribution. The three Syn KO genotypes responded to the GABA_B_R agonist/antagonist challenge with changes in the Pr and RRP that were superimposable to those observed in WT neurons (Figure 5D).

**Figure 5:** Presynaptic GABA_B_R activity similarly affects Pr and RRP size in WT, Syn I KO, Syn II KO and Syn TKO hippocampal excitatory autapses **(A)** Representative recordings evoked using high frequency stimulation (60 stimuli at 40 Hz) in autaptic neurons pretreated for 10 min with vehicle (black trace), baclofen (blue trace), GABA (1 μM; gray) or CGP55845 in the presence of 1 μM GABA (red trace). All stimulation artifacts were blanked. **(B)** Representative cumulative profiles of eEPSC amplitude for the cells shown in A. Data points in the 0.5-1.4 s window were fitted by linear regression and back extrapolated to time 0 (dashed lines) to estimate the RRP size. **(C)** Mean (± sem) values of the first current pulse of the train, RRP size and Pr for synchronous release estimated in WT autapses. For each bar, the superimposed symbols represent individual values before and after the treatments (Bclf n=8, CGP n=6; two-tailed paired Student's *t*-test with ^*^p<0.05, ^**^p<0.01, ^***^p<0.0001). **(D)** Estimation of the changes in quantal parameters induced by manipulations of GABA_B_Rs in Syn I KO, Syn II KO and Syn TKO autapses under the same conditions of panel C (Syn I KO: Bclf n= 9, CGP n=12; Syn II KO: Bclf n= 9, CGP n=6; Syn TKO: Bclf n= 9, CGP n=10; two-tailed paired Student's *t*-test with ^*^p< 0.05, ^**^p< 0.01, ^***^p< 0.0001).

### The lack of stimulation of presynaptic GABA_B_R by extracellular GABA directly contributes to the strong depression of glutamatergic transmission in TKO neurons

After the demonstration that Syn KO excitatory terminals are under the control of functional presynaptic GABA_B_Rs, we attempted to reproduce in primary autaptic cultures the facilitation/depression pattern observed ex-vivo in acute hippocampal slices of WT and TKO mice. Since excitatory autapses are characterized by a higher Pr and therefore experience a more intense response to high frequency stimulation than excitatory synapses in brain slices, depression was induced by a repetitive stimulation at 8 Hz lasting 20 s (Figure 6A). Under basal conditions, both WT and TKO synapses experienced a profound depression after a modest and transient phase of early facilitation. Depression was significantly faster in TKO neurons. Indeed after 0.5 s, the depression was significantly higher in TKO neurons (Figure 6B, right panel), while after 20 s the steady-state level was similar to that reached by WT neurons (Figure 6B, left panel).

**Figure 6:** The enhancement of synaptic depression in TKO autaptic neurons is suppressed by GABA_B_R activation **(A)** Representative eEPSCs evoked by high frequency stimulation (160 stimuli at 8 Hz) in WT and TKO hippocampal autaptic neurons. Pulse currents were superimposed to better appreciate synaptic depression. Currents are represented without artifact for clarity. **(B-F)** Time course (left) and quantitative analysis of the percentage of depression (right) in WT (black s) and TKO (red) excitatory autapses under control conditions (B) or in the presence of CGP55845 (C), baclofen (D), GABA (E) and GABA+CGP55845 (F). Quantitative analysis was carried out by measuring the first eEPSC 0.5 s after the peak of facilitation (I_p_) and 5 s after the start of the train stimulation (I_5 s_), according to the formula: (I_p_-I_5 s_)/I_p_^*^100 (see panel B). Vehicle (B): WT n=24, TKO n=29; CGP (C): WT n=9, TKO n=9; Bclf (D): WT n=5, TKO n=9; GABA (E): WT n=14, TKO n=6; CGP in GABA: WT n=11, TKO n=6. Data were analyzed by unpaired Student's *t*-test/Mann-Whitney's *U*-test; ^**^p<0.01.

Notably, WT excitatory autapses under basal conditions behave strikingly differently from WT excitatory synapses of hippocampal slices, showing synaptic depression rather than facilitation. To explain this apparent discrepancy, we challenged GABA_B_Rs with baclofen, GABA or CGP55845 to determine which of the treatments can mimic the brain slice conditions. Application of CGP55845 in the absence of exogenous GABA (Figure 6C) left the depression profiles of both WT and TKO autapses totally unaffected, confirming that in the extremely low-density culturing conditions used for growing autaptic neurons GABA spillover from the few GABAergic neurons and endogenous GABA levels in the medium are negligible. However, when either baclofen (Figure 6D) or low concentrations of exogenous GABA (1 μM; Figure 6E) were added to activate GABA_B_Rs, the depression was virtually abolished in both genotypes (Figure 6D), recapitulating the facilitation observed in WT slices in response to sustained high frequency stimulation (see Figure 2). Notably, the addition of CGP55845 after pretreatment with exogenous GABA reestablished the strong depression present under basal conditions in both WT and TKO neurons (Figure 6F).

The comparison between hippocampal slices and autaptic neurons strongly indicates that while both WT and TKO autaptic excitatory neurons are exposed to very low or null concentrations of extracellular GABA, WT pyramidal neurons in slices are exposed to a tonic GABA stimulation of presynaptic GABA_B_Rs that lowers the Pr and makes them “facilitating synapses”. On the contrary, the very low levels of extracellular GABA in TKO mice due to the impaired inhibitory transmission maintain TKO pyramidal neurons under a condition of increased Pr, due to silent GABA_B_Rs that causes the strong depressive behavior. Notwithstanding the depleted SV reserve pool of TKO terminals, this depressive phenotype was however reversible, as both WT and TKO autaptic neurons exposed to physiological concentrations of extracellular GABA or challenged with a GABA_B_R agonist switched depression into mild facilitation (Figure 6D, 6E).

In summary, our results in acute slices and autaptic neurons (see Figures 2B, and 6B, 6F, respectively) demonstrate that the lack GABA_B_R-mediated presynaptic inhibition caused by the impaired GABA release from inhibitory synapses, worsens depression of TKO excitatory synapses, exacerbating the direct effects of defective SV trafficking directly caused by Syn deletion.

## DISCUSSION

Mutations in the *SYN1* and *SYN2* genes are associated with epilepsy and/or ASD [10, 11, 12, 16] and the identification of the pathogenic mechanisms leading to the overt clinical manifestations is fundamental to establish personalized therapies. Syn I KO, Syn II KO and TKO mice are reliable experimental models of the human disease as they develop epilepsy starting from 2-3 months after birth and display an ASD-like behavior [5, 17, 18]. Previous studies in TKO autaptic neurons revealed the existence of an impairment in basal GABAergic transmission associated with a normal glutamatergic strength that was however remarkably sensitive to depression following high frequency stimulation [4]. Subsequent studies performed in hippocampal slices, revealed a striking E/I imbalance contributed by a decreased inhibitory strength and increased excitatory strength [23].

While a primary impairment of inhibitory strength was previously reported in Syn I KO neurons [19, 20], the increased excitatory strength in synapses depleted of SVs was difficult to explain. In this paper, we considered the possibility that the hyperactivity of glutamatergic transmission is a secondary heterosynaptic result of the impairment in inhibitory transmission. Under the conditions used to reveal the potentiation of glutamatergic synapses, i.e. in the presence of bicuculline [23], the decreased drive of fast GABAergic inhibition is not involved in this synaptic effect. An alternative possibility is represented by an involvement of the inhibitory control exerted by metabotropic GABA_B_Rs on glutamate release at the presynaptic level. GABA_B_Rs are located both postsynaptically and presynaptically and transduce the inhibitory action of GABA through Gβγ-mediated inhibition of voltage-gated Ca^2+^ channels and activation of K^+^ channels that shunt the action potential and further decrease Ca^2+^ influx (see [30, 31] for review). Presynaptic GABA_B_Rs are often detected extrasynaptically in glutamatergic and, to a lesser extent, GABAergic axon terminals [26]. While the preferential association of GABA_B_Rs with glutamatergic synapses suggests an important role in the regulation of excitatory synaptic strength, their frequent extrasynaptic location makes them a physiologically important target also for tonic GABA spillover, in addition to extrasynaptic GABA_A_Rs [31].

The intracellular signaling linked to GABA_B_Rs present on glutamatergic terminals is particularly critical in the inhibitory control of glutamate release and network excitability. The main effect of the stimulation of these receptors by endogenous GABA is a decrease of presynaptic Ca^2+^ influx that markedly decreases Pr [27, 30, 31, 36]. Such decrease in Pr will decrease the number of released quanta in response to single action potentials, decreasing the eEPSC amplitude and, at the same time, enhancing the response to high frequency stimulation by favoring facilitation over depression and transforming the synapse from a low to a high band-pass activity filter [33, 37]. In addition to the predominant changes in Pr, we have shown that a decreased RRP size also contributes to the presynaptic inhibition induced by GABA_B_R activation, in agreement with previous findings [28]. The latter effect, likely due to decreased SV availability or SV priming, may be mediated by the inhibition of adenylyl cyclase [27, 38] or by a decreased activation of CaM kinases I/II during high frequency activity as a consequence of the reduced Ca^2+^ influx [1].

Quantal analysis performed in WT and Syn KO autaptic excitatory neurons demonstrated that the low Pr and facilitating behavior typical of excitatory synapses mostly rely on the presence of a tonic activation of GABA_B_Rs by extracellular GABA, and that the occupancy of presynaptic GABA_B_Rs can induce fluctuations in Pr from low to high states affecting synaptic strength an short-term plasticity. We show here that the increased strength and propensity for depression observed in excitatory synapses of Syn TKO acute hippocampal slices results, at least in part, from the lack of presynaptic inhibition by GABA_B_Rs. In the absence of presynaptic GABA_B_ tone, both WT and TKO excitatory synapses experience high frequency depression. However, depression is faster and more pronounced in TKO synapses, likely because of the impaired RRP refilling due to the marked SV depletion [4, 39]. However, stimulation of GABA_B_Rs in Syn KO neurons can completely rescue the depressing phenotype, by switching high frequency depression to facilitation and overcoming the impairment in the SV supply.

The expression and synaptic responses of presynaptic GABA_B_Rs are often decreased in the hippocampus and cortical areas of epileptic patients (see [32] for a recent review). In addition, downregulation of presynaptic GABA_B_Rs associated with a reduced GABA autoinhibition has been observed in several experimental models of epilepsy, including hippocampal kindling and absence seizures [40–43]. Consistently, GABA_B_R KO mice display generalized seizures [44] and GABA_B_R antagonists are pro-epileptogenic [45]. Asynchronous GABA release, GABA spillover and tonic inhibition are known to modulate the input-output behavior of single neurons by shunting excitatory currents and hyperpolarizing the membrane potential and therefore have a protective role in epilepsy [46, 47]. A decrease in tonic inhibition was identified in some animal models of epilepsy (see [48, 49] for review), including Syn II KO and TKO mice [22, 23]. The protective role of tonic inhibition from hyperexcitability is further strengthened by the tonic stimulation of presynaptic GABA_B_Rs by extracellular GABA. In fact, stimulation of GABA_B_Rs is thought to require temporal and spatial summation of GABA released by populations of interneurons [50].

It has been reported that a fraction of glutamatergic neurons co-release GABA [33, 51]. Although corelease of GABA and glutamate is frequently observed in dentate gyrus (DG) granule cells projecting to the CA3 region, but not in the Schaffer collateral-CA1 synapses, co-released GABA by excitatory terminals can participate in the GABA_B_R-mediated regulation of excitatory strength and short-term plasticity. At the moment, it is not clear whether corelease involves distinct pools of SVs with different Ca^2+^ sensitivities, and therefore it is difficult to evaluate the impact of Syn deletion on glutamate/GABA corelease. However, the decreased extracellular GABA and tonic current observed in hippocampal slices of both TKO mice [23] and SynII KO mice [22] indicates that, no matter of single release or corelease, glutamatergic and GABAergic transmissions are differentially affected by Syn deletion.

These findings, together with the previous data on single Syn I and Syn II KO mice, allow depicting a hyperexcitability/epileptogenesis pathway in TKO mice. It has been found that lack of Syn I decreases synchronous GABA release [19, 20], while lack of Syn II markedly impairs asynchronous GABA release [21]. It was subsequently demonstrated that both Syn II KO and TKO mice have an extremely low tonic current and that this current is greatly contributed by the spillover of asynchronously released GABA [22, 23]. This primary impairment in GABA transmission is followed by an increased intrinsic excitability of glutamatergic neurons by impairment of phasic inhibition and lack of tonic GABA_A_R-mediated shunting inhibition. However, the low extracellular levels of spilled over GABA also leave presynaptic GABA_B_Rs unoccupied, with a resulting lack of the homeostatic presynaptic inhibitory brake on evoked glutamate release. These findings allow identifying the impairment in GABA release as the *primum movens* of the hyperexcitability of Syn KO mice. Since the extent of inhibition provides stability to neuronal networks, such imbalance may force neuronal circuits into a state of heightened excitability that triggers epileptogenesis, resulting in the late (2-3 months of age) appearance of the overt epileptic phenotype in mice bearing Syn gene deletion [2–5] and in man with loss-of-function mutations in *SYN* genes [15]. A possible pathogenetic pathway for the E/I imbalance in TKO neurons and the respective contributions of the single Syn gene products are schematically shown in Figure 7. The summation of the specific effects arising from the lack of Syn I and Syn II explain why, even in the absence of redundant functions of the two isoforms on neurotransmitter release dynamics, the epileptic phenotype of TKO mice is more severe that those of single KO mice.

**Figure 7:** Schematics of the possible pathogenic pathway for the E/I imbalance in Syn TKO neurons Deletion or loss-of-function of *SYN* genes causes a primary impairment of synchronous and asynchronous GABA release due to the defective recruitment and priming of SVs. The resulting defect in phasic and tonic inhibition in turn generates E/I imbalance that increases network excitability. At the same time, the decreased GABA spillover leaves presynaptic GABA_B_Rs unoccupied, resulting in inactivation of the inhibitory brake on glutamate release and an increased strength of excitatory transmission that worsens the E/I imbalance and triggers epileptogenesis.

The clarification of the epileptogenic pathway in Syn KO mice identifies important targets for pharmacological treatments to cure epilepsy in patients bearing *SYN* mutations. According to this interpretation, the combined administration of extrasynaptic GABA_A_R agonists such as gaboxadol [22] and GABA_B_R agonists such as baclofen should attenuate the E/I imbalance of TKO networks by regaining control on both excitability and synaptic strength of excitatory neurons. As the E/I imbalance is observed well before the onset of seizures, a preventive treatment with these drugs not impacting directly on fast inhibition could potentially dampen epileptogenesis and abort/prevent the resulting epileptic phenotype.

## MATERIALS AND METHODS

### Materials

#### Mice

Homozygous Syn TKO mice [4] were kindly provided by Drs. H-T. Kao (Brown University, Providence, RI) and Paul Greengard (The Rockefeller University, NY). TKO mice were re-derived on a C57BL/6J background (Charles River, Calco, Italy), obtaining single and multiple Syn KO strains up to the triple Syn knockout (TKO) and matched wild type (WT) mice. One-month-old mice of either sex were used. All experiments were carried out in accordance with the guidelines established by the European Community Council (Directive 2010/63/EU of September 22nd, 2010) and were approved by the National Council on Health and Animal Care (authorization ID 227, prot. 4127 25th March 2008).

#### Drugs

Bicuculline methiodide (30 μM) and (2R)-amino-5-phosphonovaleric acid; (2R)-amino-5-phosphonopentanoate (APV; 100 μM) were applied to isolate AMPA receptor-dependent eEPSCs. CGP55845 (5 μM) or Baclofen (20 μM) was applied to study the effect of GABAB receptor blockade/activation. All drugs were purchased from Tocris Bioscience (Bristol, UK). Cell culture media were from Invitrogen. All other chemicals were from Sigma.

### Electrophysiology in acute hippocampal slices

#### Tissue preparation

Hippocampal slices were prepared as previously described [23]. Mice were anaesthetized with halothane (Sigma-Aldrich, Milan, Italy) and decapitated; the brain was quickly removed and immersed in an ice-cold “cutting” solution composed of (mM): 125 NaCl, 25 NaHCO_3_, 25 glucose, 2.5 KCl, 1.25 NaH_2_PO_4_, 1 CaCl_2_, 2 MgCl_2_, 0.4 Ascorbic acid, 2 NaPyruvate, 3 *myo*-Inositol and saturated with 95% O_2_ and 5% CO_2_. Horizontal hippocampal slices (250 μm-thick) were cut using a HM 650 vibratome (Microm International GmbH, Walldorf, Germany) in ice-cold oxygenated “cutting” solution. Slices were first incubated in “cutting” solution at 35 °C for 30 min and then transferred to a “submerged” recording chamber in a “standard recording” solution composed of (mM): 125 NaCl, 25 NaHCO_3_, 25 glucose, 2.5 KCl, 1.25 NaH_2_PO_4_, 2 CaCl_2_, 1 MgCl_2_. This solution was constantly oxygenated, maintained at 33 °C and superfused at a rate of 1.5 ml/min.

#### Electrophysiological recordings

Whole-cell voltage-clamp recordings from CA1 pyramidal neurons of hippocampal slices were performed with glass pipettes (~3.8 to 5 MΩ) pulled from borosilicate glass (Kimble Glass Inc., Vineland, NJ) and filled with the following intracellular solution (mM): 126 Kgluconate, 4 NaCl, 1 MgSO_4_, 0.02 CaCl_2_, 0.1 BAPTA, 15 glucose, 5 HEPES, 3 ATP, 0.1 GTP. Pyramidal neurons of CA1 region of the hippocampus were visualized with a 40X water immersion objective and an infrared camera. Voltage-clamp recordings were conducted at the holding potential of -70 mV and data were acquired using the MultiClamp 700B amplifier and the pClamp 9.2 software (Axon Instruments, Molecular Devices, Sunnyvale, CA). The acquisition frequency was 10 kHz and the filter used was 2 kHz; series resistance was monitored throughout the experiment and whenever it changed more than 15%, the recording was not included in the analysis. eEPSCs were evoked in pyramidal neurons by electrical stimulation of Schaffer collaterals with a bipolar tungsten electrode (test pulses at 0.1 Hz, 0.25 ms duration). For single pulse responses, the stimulus intensity was varied from the lowest intensity able to evoke eEPSCs to an intensity eliciting the maximum current amplitude. For the short-term plasticity recordings, the stimulation was adjusted at intensity able to evoke 2/3 of the maximum eEPSC amplitude for synaptic depression and recovery the baseline was evaluated as the mean eEPSC amplitude during 5 min of stimulation at 0.1 Hz. The high frequency repetitive stimulation protocol (20 Hz for 20 s) was applied and followed by lower stimulation frequency (0.1 Hz) to evaluate the rate and extent of recovery from synaptic depression. Each cell was normalized to the mean baseline value and averaged with other cells, Electrophysiology in hippocampal autapses

#### Preparation of hippocampal autaptic cultures

Mice were sacrificed by inhalation of CO_2_, and 17/18-day embryos (E17-E18) were removed immediately by cesarean section. Removal and dissection of hippocampi were previously described [52]. Briefly, hippocampi were dissociated by enzymatic digestion in 0.125% Trypsin for 20 min at 37 °C and then triturated with a fire-polished Pasteur pipette. No antimitotic drugs were added to prevent glia proliferation. Autaptic neurons were prepared as described previously [35] with slight modifications. Dissociated neurons were plated at very low density (20 cells/mm^2^) on microdots (40-300 μm in diameter) obtained by spraying a mixture of poly-D-lysine (0.1 mg/ml) and collagen (0.25 mg/ml) on dishes that had been pretreated with 0.15% agarose. Both glial cells and single autaptic neurons were present under this culture condition.

#### Patch-clamp recordings, data acquisition and analysis

Whole-cell patch-clamp recordings were made from autaptic neurons grown on microislands, as previously described [19, 53]. Patch electrodes, fabricated from thick borosilicate glass (Hilgenberg, Mansfield, Germany), were pulled to a final resistance of 3-4 MΩ. eEPSCs were recorded using an EPC-10 amplifier (HEKA Electronic, Lambrecht, Germany) by superfusing the whole-cell clamped neuron with a Tyrode solution containing (in mM): 140 NaCl, 2 CaCl_2_, 1 MgCl_2_, 4 KCl, 10 glucose,10 HEPES (pH 7.3 adjusted with NaOH). D-(-)-2-amino-5-phosphonopentanoic acid (D-AP5; 50 μM; Tocris, Bristol, UK) was added to the Tyrode solution to block N-methyl-D-aspartate receptors, respectively. The standard internal solution was (in mM): 126 K gluconate, 4 NaCl, 1 MgSO_4_, 0.02 CaCl_2_, 0.1 BAPTA, 15 glucose, 5 HEPES, 3 ATP, 0.1 GTP (pH 7.2 adjusted with KOH). All the experiments were performed at room temperature. Neurons were voltage clamped at -70 mV. Action potentials were evoked by depolarizing the cell body to +40 mV for 0.5 ms at 0.1 Hz. eEPSCs were acquired at 10-20 kHz and filtered at one fifth of the acquisition rate with an 8-pole low-pass Bessel filter. Recordings with leak currents >100 pA or series resistance >10 MΩ were discarded. Data acquisition was performed using PatchMaster programs (HEKA Elektronic, Lambrecht, Germany). eEPSCs were inspected visually, and only those that were not contaminated by spontaneous activity were considered. To calculate the peak current during an isolated stimulus or a train of stimuli, we first subtracted an averaged trace containing the stimulus artifact and the action potential current, but lacking any discernable synaptic current (i.e. synaptic failures). Such traces were easily identified toward the end of a train of stimuli, when synaptic depression was maximal. These traces were averaged and scaled to the peak Na^+^ current contaminating the eEPSC.

To analyze PPR, two brief supraliminar depolarizing pulses were applied to autaptic neurons at 50 ms intervals. For each couple of eEPSCs, PPR was calculated as the ratio I_2_/I_1_, where I_1_ and I_2_ are the amplitudes of the eEPSCs evoked by the conditioning and test stimuli, respectively. The amplitude of I_2_ was determined as the difference between the I_2_ peak and the corresponding value of I_1_ calculated by mono-exponential fitting of the eEPSC decay [54]. Because of the high intrinsic variability of PPR, the mean PPR was calculated from the responses to at least 4-8 paired-pulse stimulation protocols for each interpulse interval.

#### Cumulative eEPSC amplitude analysis

The size of the RRP and Pr were calculated using the cumulative amplitude analysis [19]. RRP was determined by summing up peak eEPSC amplitudes during 40 repetitive stimuli applied at 40 Hz. This analysis assumes that depression during the steady-state phase is limited by a constant recycling of SVs and an equilibrium occurs between released and recycled SVs [55, 56]. The number of data points for the linear fitting of the steady-state phase was evaluated by calculating the best linear fit including the maximum number of data points starting from the last one (i.e., from the 40^th^ eEPSC). The intercept with the Y-axis gave the RRP and the ratio between the amplitude of the first eEPSC (I_1_) and RRP yielded the Pr.

### Statistical analysis

Data are expressed as means ± sem for number of cells (n). Normal distribution of data was assessed using D’Agostino-Pearson's normality test. The F-test was used to compare variance between two sample groups. To compare two normally distributed sample groups, the Student's unpaired or paired *t*-test was used. When two sample groups were not normally distributed, the non-parametric Mann-Whitney's *U*-test was used. To compare more than two normally distributed sample groups, one-way ANOVA, followed by post-hoc multiple comparison tests was used. Alpha levels for all tests were 0.05% (95% confidence intervals). Statistical analysis was carried out using OriginPro-8 (OriginLab Corp., Northampton, MA, USA) and Prism (GraphPad Software, Inc.) software.

## Abbreviations

ASD: autism spectrum disorder
CGP55845: (2S)-3-[[(1S)-1-(3,4-dichlorophenyl) ethyl] amino-2-hydroxypropyl] (phenylmethyl) phosphinic acid
E/I: excitation/inhibition
DG: dentate gyrus
eEPSC: evoked excitatory postsynaptic current
GABA: γ-aminobutyric acid
GABA_B_R: GABA_B_ receptor
KO: knockout
PPR: paired-pulse ratio
Pr: probability of release
RRP: readily releasable pool for synchronous release
SV: synaptic vesicle
Syn: synapsin
TKO: triple knockout
WT: wild type
